# Mild Hypothermia Therapy Lowers the Inflammatory Level and Apoptosis Rate of Myocardial Cells of Rats with Myocardial Ischemia-Reperfusion Injury via the NLRP3 Inflammasome Pathway

**DOI:** 10.1155/2021/6415275

**Published:** 2021-08-09

**Authors:** Renjun Gao, Hongye Zhao, Xianyan Wang, Bo Tang, Yu Cai, Xinrui Zhang, Hao Zong, Yitong Li, Yanli Wang

**Affiliations:** ^1^The Sixth Department of Cardiology, The Second Affiliated Hospital of Qiqihar Medical University, Qiqihar, Heilongjiang 161006, China; ^2^Department of Physiology, Qiqihar Medical University, Qiqihar, Heilongjiang 161006, China; ^3^Department of Pathology, Qiqihar Medical University, Qiqihar, Heilongjiang 161006, China

## Abstract

**Objective:**

To explore the protective effects and mechanism of mild hypothermia treatment in the treatment of myocardial ischemia-reperfusion injury. *Material and Methods*. A total of 20 Sprague-Dawley (SD) rats were assigned to 4 groups: the blank control group, sham operation group, ischemia reperfusion group, and mild hypothermia therapy group (each *n* = 5). Some indexes were detected. In addition, myocardial cell models of oxygen-glucose deprivation/reoxygenation injury (OGD) were established. The expression of mRNA IL-6 and TNF-*α* and the key enzyme levels of apoptosis (cleaved-Caspase-3) and the NLRP3 inflammasome/p53 signaling pathway in the models were determined.

**Results:**

The expression of serum IL-6 and TNF-*α* in the mild hypothermia therapy group was significantly lower than that in the ischemia reperfusion group. The mild hypothermia therapy group also showed a significantly lower TUNEL cell count and NLRP3 and p53 phosphorylation levels than the ischemia reperfusion group (all *p* < 0.05). The in vitro mild hypothermia + OGD group also showed significantly lower mRNA expression of IL-6 and TNF-*α* and levels of cleaved Caspase-3, NLRP3, and phosphorylated p53 protein than the OGD group (all *p* < 0.05).

**Conclusion:**

In conclusion, mild hypothermia therapy can inhibit the apoptosis and myocardial inflammation of cells induced by MI/R injury in rats and inhibiting the activity of the NLRP3 inflammasome pathway and p53 signaling pathway may be the mechanism.

## 1. Introduction

Cardiovascular diseases are the leading cause of death in the world, which accounts for 25% of all causes of death worldwide in 2010 and 31% of all causes of death worldwide in 2016, and 85% cardiovascular disease-related deaths are caused by heart attack and stroke [1]. In China, cardiovascular diseases also occupy the first place in the cause of death, accounting for about 40% of all causes of death. As a country with a large population, China is one of the countries with the heaviest medical burden for cardiovascular diseases in the world [2]. Acute myocardial infarction (AMI) is a myocardial necrosis event caused by unstable myocardial blood supply and is a primary cause of heart attack and stroke [3]. The pathophysiological mechanism of AMI is as follows: chronic atherosclerosis gives rise to coronary stenosis and atherosclerotic plaque disruption and then causes plaques out from platelets that participate in blood circulation, resulting in the hypercoagulable state of blood vessels and rupture of other unstable plaques through feedback triggering, which eventually leads to irreversible necrosis of myocardial cells. At present, AMI is treated mainly by restoring the blood flow in time (including thrombolytic therapy, percutaneous coronary intervention, and coronary artery bypass graft) and reducing the myocardial infarction area [4]. Although surgical treatment and drug therapy can restore blood flow in time and greatly reduce the mortality of patients with AMI, there are still 25% patients who develop heart failure or even die [5, 6].

Mild hypothermia therapy is an intervention method to control the patient's core temperature at 32–35°C. Mild hypothermia can reduce mortality and nerve injury when used for resuscitation after cardiac arrest. In case of an out-of-hospital cardiac arrest, the International Liaison Committee on Resuscitation (ILCR) recommends that the body temperature of patients shall be cooled to 32–34°C for 12–24 hours when their cardiac rhythm recovers to initial ventricular fibrillation [7]. In recent years, the research on mild hypothermia therapy in myocardial infarction is still controversial. On one hand, some studies have found that mild hypothermia therapy can increase the cure rate of patients with out-of-hospital cardiac stroke and protect their brain function [8, 9]. On the other hand, some studies have pointed out that mild therapeutic hypothermia will not lower the mortality of heart diseases and the incidence rate of adverse cardiac events [10]. Moreover, in terms of basic research, several studies have confirmed that mild hypothermia therapy can reduce the myocardial infarction area in animal models of AMI [11].

In the preliminary clinical trials of small samples, there is no evidence that mild hypothermia therapy can take positive effect [12], but in another multicenter clinical trial of mild hypothermia therapy, it has been found that mild hypothermia therapy can reduce the myocardial infarction area [13]. A meta-analysis on mild hypothermia therapy for AMI has shown that mild hypothermia (34°C) therapy neither is conducive to the myocardial infarction area and cardiac function nor does it prolong the time required for completing the whole course of door-to-balloon and the time required for initial percutaneous coronary interventions (PCI) [14].

However, the specific role of mild hypothermia in the myocardium, including the effects of mild hypothermia on myocardial inflammation and myocardial cell apoptosis and the specific molecular mechanism, has not been fully elucidated. This study is aimed at investigating the effects of mild hypothermia therapy on myocardial inflammation and the apoptosis level of cells during myocardial infarction and its potential mechanism by simulating the pathophysiological changes of ischemia/hypoxia-reperfusion injury during myocardial infarction using rat models of myocardial ischemia-reperfusion (MI/R) injury and cultured embryonic cardiac myocytes of oxygen glucose deprivation/reoxygenation (OGD) and adopting mild hypothermia intervention for the models.

## 2. Materials and Methods

### 2.1. Research Materials

#### 2.1.1. Experimental Animals

A total of 20 Sprague-Dawley (SD) rats (200–250 g) were purchased from Hunan SJA Laboratory Animal Co. Ltd., with a license number of SCXK (Xiang) 2016-002.

#### 2.1.2. Main Reagents

Embryonic cardiac myocytes of rats (H9c2 cell lines) (Chinese Academy of Sciences), enzyme-linked immunosorbent assay (ELISA) kits for interleukin-6 (IL-6) and tumor necrosis factor-*α* (TNF-*α*) in rats (E-EL-R0015c and E-EL-R0019c, Elabscience Biotechnology Co. Ltd., Wuhan, China), DNA/RNA/protein co-extraction kit (DP423, Tiangen Biotech Co. Ltd., Beijing, China), in situ apoptosis assay kit (11684795910, Roche Group, Switzerland), kit for rapid preparation of SDS-PAGE gel (P0012AC, Beyotime Biotechnology Co. Ltd., Shanghai, China), TRIzol (15596026, Thermo Fisher Scientific, Shanghai, China), polymerase chain reaction (PCR) kit (YT379, Biolab Technology, Beijing, China), NOD-, LRR-, pyrin domain-containing protein 3 (NLRP3) antibody (ab214185, Abcam Company, USA), phosphorylated p53 (9284, CST Company, USA), Caspase-3 antibody (9662, CST Company, USA), and GAPDH antibody (ab181602, Abcam Company, USA) are the main reagents. The concentration of all antibodies was 1 : 1000.

### 2.2. Rat Models of Coronary Artery Ischemia-Reperfusion Injury-Induced AMI

In this study, rat models of MI/R injury constructed by coronary artery occlusion were adopted to stimulate AMI after being modified [15]. Rats were randomly assigned to four groups: blank control group (control group), sham operation group (sham group), ischemia reperfusion group (IRI group), and mild hypothermia therapy group (IRI + mild hypothermia) (each *n* = 5). The rats were weighted and intraperitoneally injected with pentobarbital sodium (80 mg/kg) for anesthesia. Under anesthesia, the rats were treated for skin preparation on their neck and chest and their operation sites were disinfected, followed by skin cutting on the neck. Subsequently, each rat was connected with a ventilator through tracheal intubation and was given positive pressure mechanical ventilation (tidal volume: 10 mL; ventilator frequency: 90 times; and ratio: 1 : 1). In the fourth intercostal space on the left side of the sternum of each rat, the skin was cut apart vertically and the third rib was cut off to open the thoracic cavity and expose the heart and the rat was given 200 u/kg heparin sodium before coronary artery occlusion and was given 0.5% lidocaine before ligation of the left coronary artery. Subsequently, a 6-0 nylon surgical thread was used for ligation by inserting the needle at the site about 2 mm away from the aortic root between the inferior edge of the left atrial appendage and the pulmonary artery cone by inserting about 2 mm in width and depth after threading. After successful ligation, there was a phenomenon that the anterior wall of the left ventricle became purple or pale in naked eyes, with weakened pulsation, and there was an elevation in the ST segment in the connected electrocardiogram marked myocardial ischemia, which implied the success modeling of cardiac ischemia. In the mild hypothermia group, rats were immediately placed on a temperature control device and the temperature was set at 32°C. We inserted a thermometer into the rectum to confirm that the rat's body temperature was 32°C, while rats in the ischemia reperfusion group were placed at room temperature (without body temperature intervention). The visual operative field of thoracic surgery was covered with gauze wet by normal saline. After 30 min, the ligature was cut off to form reperfusion and the color of myocardium was analyzed. Afterwards, the muscle and skin were sutured in turn and again disinfected with povidone iodine. Finally, the heart of each rate was reperfused for 1 h and the rat was killed by carbon dioxide narcosis (euthanasia), followed by collection of serum and heart tissue for subsequent detection.

### 2.3. Construction of In Vitro Myocardial Cell Models of OGD Intervened with by Mild Hypothermia

Rat-derived parent myocardial cell lines (H9c2 cell lines) were purchased form ATCC. They were cultured in high-glucose (4.5 g/L D-glucose) complete Dulbecco's modified Eagle medium (DMEM) containing fetal bovine serum (FBS) (10%) in a CO_2_ (5%) incubator at 37°C. The experimental groups consisted of 4 groups: the blank control group (control group), mild hypothermia control group (mild hypothermia group), OGD group, and OGD + mild hypothermia culture group (OGD + mild hypothermia group). In the control group, cardiomyocytes were cultured in an incubator containing high-glucose DMEM medium with 10% FBS and 5% CO_2_ at 37°C for 24 h and cardiomyocytes in the mild hypothermia group were cultured in a mild hypothermia incubator containing high glucose DMEM medium with 10% FBS and 5% CO_2_ at 32°C for 24 h. In addition, cardiomyocytes in the OGD + mild hypothermia group were cultured in DMEM medium (low glucose, 1 g/L D-glucose) containing 10% FBS. We placed these cardiomyocytes in a mild-hypothermia three-gas incubator (32°C, containing 0.5% O_2_, 5% CO_2_, and 94.5% N_2_) for 6 hours. Then, these cardiomyocytes were cultured in an incubator containing high-glucose DMEM medium with 10% FBS and 5% CO_2_ at 37°C for 24 h. The RNA was extracted from them, followed by determination of the expression of IL-6 and TNF-*α*. Proteins were extracted from the cells, and the expression of apoptosis-related cleaved Caspase-3 and Caspase-3, NLRP3 protein, phosphorylated p53 protein, and total p53 protein was determined.

### 2.4. Determination of the Levels of Serum IL-6 and TNF-*α* by ELISA

After cardiac perfusion, blood of rats was sampled through pericardiocentesis, left at room temperature for 1 hour, and centrifugated at 12000 g·rpm for 5 min to collect serum. The serum IL-6 and TNF-*α* were quantified, using the corresponding ELISA kits in accordance with the kit instructions. The optical density of samples was measured at 450 nm using a microplate reader to calculate the serum IL-6 and TNF-*α* expression in each group.

### 2.5. Extraction of Protein from Heart Tissue

Heart tissue (1 g) was sampled from each rat, and the protein of the tissue was extracted using the DNA/RNA/protein coextraction kit and quantified using the bicinchoninic acid (BCA) method.

### 2.6. Western Blot (WB) Assay

10% SDS-PAGE gel was prepared using the kit for rapid preparation of SDS-PAGE gel (Beyotime Biotechnology Co. Ltd., Shanghai, China), and the loading quantity of the sample protein was 20 *μ*g. The sample protein was subjected to electrophoresis at 80 V for 30 min, followed by electrophoresis at 120 V for 1 h. Subsequently, the protein was transferred to a PVDF membrane through the wet transfer method at a constant current of 350 mA for 1 h and the membrane was blocked in 5% skim milk/TBST at room temperature for 1 h and washed with TBST and the antibody and GAPDH (internal reference control) were diluted by 5% defatted milk at 1 : 1000 and then incubated at 4°C overnight. Afterwards, the membrane was washed with TBST and incubated with corresponding secondary antibody (goat anti-rabbit (1 : 1000) and goat anti-mouse (1 : 5000)) at room temperature for 1 h. Finally, the intensity of corresponding protein was detected by the electrochemiluminescence (ECL) method after TBST washing. The band intensity was analyzed using the ImageJ software (NIH, USA).

### 2.7. TUNEL Staining of Paraffin Sections of Myocardial Tissue

Myocardial tissue was fixed with 10% paraformaldehyde and embedded in paraffin. The paraffin-embedded tissue blocks of myocardium were cut into 4 *μ*m thick sections, and in situ cell apoptosis was detected using staining according to the terminal deoxynucleotidyl transferase-mediated dUTP nick-end labeling (TUNEL) kit instructions. The number of TUNEL-positive cells in each group of myocardial sections was analyzed under an immunofluorescence microscope and compared.

### 2.8. RNA Extraction and Common PCR/Agarose Gel Electrophoresis

RNA of cells was extracted using TRIzol [16], and the RNA was reversely transcribed into cDNA using the PCR kit. The PCR reaction conditions were 94°C 3 min, 94°C 15 sec, and 60°C 30 sec. Forty cycles of reactions were carried out on the StepOnePlus Detection System (ABI, USA), and the 2 − △△*CT* method was used to calculate the gene expression. The primer sequences used were as follows: IL-6 primer sequence (upstream primer: CCACCCACAACAGACCAGTA-3′; downstream primer: 5′-GGAACTCCAGAAGACCAGAGC-3′); TNF-*α* primer sequence (upstream primer: 5′-ACGTCGTAGCAAACCACCAA-3′; downstream primer: 5′-AAATGGCAAATCGGCTGACG-3′); *β*-actin primer sequences (upstream primer: 5′-TCAGGTCATCACTATCGGCAAT-3′; downstream primer: 5′-AAAGAAAGGGTGTAAAACGCA-3′). All primers were synthesized by Thermo Fisher Scientific (Shanghai).

### 2.9. Statistical Analysis

Experimental data were analyzed by SPSS20.0. Comparison between groups was analyzed by ANOVA followed by TUKEY. *p* < 0.05 indicates a significant difference.

## 3. Results

### 3.1. Mild Hypothermia Therapy Lowers the Levels of Serum Inflammatory Factors in Rat Models of AMI

The serum expression of inflammatory factors IL-6 and TNF-*α* was detected by ELISA (Figure 1). In the ischemia reperfusion group (IRI), the levels of serum IL-6 and TNF-*α* of AMI were significantly higher than those in the control group (control) and the sham group (sham), and IL-6 and TNF-*α* levels in the mild hypothermia group (IRI + mild hypothermia) were significantly lower than those in the ischemia reperfusion group (IL-6, *p* = 0.0001; TNF-*α*, *p* = 0.0071).

### 3.2. Mild Hypothermia Intervention Weakens the Myocardial Apoptosis of Rat Models of AMI

The TUNEL was adopted to determine the apoptosis level of myocardial cells in rat models of AMI. In Figure 2, myocardial apoptosis was rare in the control group and the sham group (cells labeled with green fluorescence were apoptotic cells), while the myocardial apoptosis count in the ischemia reperfusion group significantly increased (Figure 2(a)). In the mild hypothermia group, the number of apoptotic cells was significantly lower than that in the ischemia reperfusion group (*p* < 0.0001, Figure 2(b)).

### 3.3. Mild Hypothermia Regulates the Myocardial Inflammation and Apoptosis by Inhibiting the Inflammasome NLRP3/p53 Signaling Pathway

In order to further investigate the regulatory mechanism of mild hypothermia therapy on the inflammation level and myocardial cell apoptosis of rats with myocardial infarction, we detected the expression level of NLRP3 protein and the phosphorylation level of p53 molecule in myocardial tissue inflammasome by a WB assay. As shown in Figure 3, in the ischemia reperfusion group, the phosphorylation levels of NLRP3 and p53 in the myocardial tissue were significantly higher than those of the control group and the sham group, while the phosphorylation levels of NLRP3 and p53 in the mild hypothermia group were significantly lower than those of the ischemia reperfusion group (NLRP3: *p* = 0.0019; p53: *p* = 0.0016).

### 3.4. Mild Hypothermia Inhibits the Inflammation Level of In Vitro Myocardial Cell Models of OGD

In order to further explore the effects of mild hypothermia on myocardial cells, we constructed in vitro cultured myocardial cell models of OGD to simulate ischemia-reperfusion injury during myocardial infarction. The IL-6 and TNF-*α* mRNA expression was determined using the PCR/agarose gel method. In Figure 4, compared with the control group, the OGD group showed significantly increased mRNA expression of IL-6 and TNF-*α* (both *p* < 0.0001), and compared with the OGD group, the OGD + mild hypothermia group showed significantly decreased mRNA expression of IL-6 and TNF-*α* (IL-6: *p* = 0.0037; TNF-*α*: *p* = 0.0007).

### 3.5. Mild Hypothermia Inhibits the Inflammatory Level and Apoptosis of In Vitro Myocardial Cell Models of OGD by Interfering with the Inflammasome NLRP3/p53 Signaling Pathway

The effects of mild hypothermia were reflected by the level changes of cleaved Caspase-3/Caspase-3 protein after OGD of in vitro myocardium. As shown in Figure 5(a), the WB assay revealed that the cleaved Caspase-3/Caspase-3 ratio in the OGD group was significantly higher than that in the mild hypothermia group and the control group, but significantly lower than that of the OGD + mild hypothermia group (*p* = 0.0172).

To further investigate the mechanism of mild hypothermia in regulating myocardial cell apoptosis and the inflammatory level, we explored the expression of the inflammasome NLRP3/p53 signaling pathway in myocardial cell models of OGD. As shown in Figure 5, the phosphorylation levels of NLRP3 protein and p53 protein in the OGD group were significantly higher than those in the mild hypothermia group and the control group and their phosphorylation levels were significantly lower in the mild hypothermia + OGD group than those in the OGD group (*p* < 0.0001).

## 4. Discussion

At present, mild hypothermia therapy has definite neuroprotective effect on patients in resuscitation but its clinical advantages for AMI are still under investigation. In the preliminary clinical trials of small samples, there is no evidence that mild hypothermia therapy can reduce adverse cardiovascular events [12]. A meta-analysis on mild hypothermia therapy for AMI has shown that mild hypothermia (34°C) therapy is not conducive to the myocardial infarction area and cardiac function nor does it prolong the time required for completing the whole course of door-to-balloon and the time required for initial percutaneous coronary interventions (PCI) [14]. However, it has been found in another multicenter clinical trial of mild hypothermia therapy that mild hypothermia therapy can reduce the myocardial infarction area [13] and mild hypothermia therapy can exert cardiac protection effect only on the ischemic period and there is no evidence that it can exert positive effects on the reperfusion period [17]. The difference in clinical advantages of mild hypothermia therapy may be due to the different target temperatures used in various studies and the different cooling methods used, which makes it difficult to control the core temperature of patients at 32–35°C without changes. Another reason may be that there are some mechanisms that limit the effect of mild hypothermia therapy. For example, subgroup analysis of clinical trial patients shows that anterior myocardial infarction is significantly smaller than myocardial infarction in other parts after mild hypothermia therapy [10]. Therefore, the effects of mild hypothermia therapy on AMI need to be further explored.

Previous studies have revealed that mild hypothermia intervention has protective effect on organs against ischemia-reperfusion injury. For example, mild hypothermia therapy can alleviate inflammatory response in rat models of ischemia-reperfusion injury [18] and it can exert stronger protective effect on the liver of obese rats than thin rats [19]. Mild hypothermia therapy is well studied in cerebral ischemic injury. Low temperature can alleviate the oxidative stress injury induced by hypoxia/reoxygenation of the cerebral vascular barrier (human brain microvascular endothelial cells, stellate cells, and peripheral cells) simulated by in vitro culture and enhance the antioxidant capacity [20], and it can also inhibit the accumulation of glutamate, a mediator of excitotoxic brain injury, reduce the generation of oxygen free radicals, and weaken neuron apoptosis and cell autophagic death by reducing the generation of apoptosis-promoting proteins such as p53 protein, Bax, Bak, and NAD [21]. As for the heart, some researchers have used 34°C to interfere with rat models of left coronary artery ischemia-reperfusion injury and treated the models with ischemia for 30 minutes and reperfusion for 24 hours. It turned out that mild hypothermia intervention can reduce the myocardial infarction area and neutrophil infiltration and may reduce myocardial cell apoptosis [22] and increase autophagy flow in myocardial cells, mitochondrial autophagy, and mitochondrial quality to alleviate the myocardial fibrosis degree [23]. The cardioprotective effect of mild therapeutic hypothermia is not only to reduce the myocardial infarction area but also to protect the myocardial contractile function after ischemia, prevent microvascular circulation without reflux occlusion, and prevent left ventricular remodeling [24]. The molecular mechanism of mild hypothermia is not only to inhibit cell metabolic consumption but also to activate protective cell signal transduction pathways, such as the Akt/ERK1/2 signaling pathway and the PI3K/mTOR signaling pathway [24, 25]. Despite the in-depth research on the abovementioned signaling pathways, it is found that a single Akt inhibitor or mTOR inhibitor still has limited myocardial protection and more upstream-specific signaling mechanisms need to be found in order to better cooperate with the clinical application of mild hypothermia therapy.

Cardiac ischemia-reperfusion injury is an important pathophysiological change during myocardial infarction. Previous studies have mostly considered oxidative stress, calcium overload, vascular endothelial injury, and myocardial cell apoptosis as mechanisms of further myocardial injury caused by the MI/R process [20, 26–28]. In recent years, it has become a research hotspot to alleviate myocardial infarction injury by intervening with myocardial cell apoptosis. NLRP3 is an intracellular receptor that forms and activates NLRP3 inflammasome after receiving microbial signals, exogenous danger signals, and environmental stress signals. The assembly and activation of NLRP3 inflammasome lead to the release of Caspase-1-dependent proinflammatory factors (IL-1*β* and IL-18) and can also induce cell apoptosis mediated by protein gasdermin D [29]. The role of NLRP3 inflammasome in MI/R injury has been widely studied, but it is still controversial. On one hand, some studies have found that NLRP3 is upregulated in rat models of myocardial ischemia reperfusion [30], and the NLRP3 inflammasome level decreased by drugs can alleviate myocardial injury [31]. In addition, it has been found that NLRP3 inflammasome is activated in rat models of diabetes mellitus, which may aggravate MI/R injury by mediating myocardial cell apoptosis [32]. NLRP3 inflammasome can interact with cellular pathways of a variety of cells, which may be the upstream effector of the Akt/ERK1/2 signaling pathway [33]. On the other hand, one study has revealed that the MI/R injury in mice with NLRP3 gene deficiency is more serious than that in wild-type mice and it is believed that NLRP3 inflammasome plays a protective role against MI/R injury [34]. In the process of aggravation of MI/R injury due to high-fat and high-fructose diet, NLRP3 inflammasome is activated, which promotes the activation of the myocardial-protective RISK/HIF-2*α* signaling pathway [35]. However, the role of NLRP3 inflammasome in MI/R injury under mild therapeutic hypothermia has not been reported.

In this study, we constructed in vivo and in vitro myocardial infarction models, AMI models induced by myocardial ischemia reperfusion, and myocardial cell models of OGD and simulated the pathophysiological changes of myocardial infarction at the animal level and cell level, respectively. We intervened with models with mild hypothermia and explored the pathophysiological process and mechanism of mild hypothermia intervention on myocardial infarction. In vivo, mild hypothermia therapy can significantly reduce myocardial TUNEL-positive cell count and serum TNF-*α* and IL-6 levels. The TNF-*α* and IL-6 mRNA expression and cleaved Caspase-3 protein expression in vitro myocardial cell models of OGD after mild hypothermia intervention were significantly lower than those in myocardial cells in the OGD model, indicating that mild hypothermia intervention had antiapoptosis and anti-inflammation effects on myocardial cells in vivo and in vitro. In order to further explore the molecular mechanism of mild hypothermia therapy on myocardial protection, we conducted a literature review from the mechanisms related to inflammation and apoptosis and found that the NLRP3 inflammasome signaling pathway plays a key role in mediating MI/R injury. Therefore, with this finding as a breakthrough point, we inferred that mild hypothermia therapy inhibited the apoptosis and inflammatory level of myocardial cells by inhibiting the NLRP3 inflammasome signaling. The detection of the protein level of NLRP3 in in vivo and in vitro models revealed that the NLRP3 level in myocardial cells was significantly increased in ischemia-reperfusion injury models and OGD models, while it was significantly decreased after mild hypothermia intervention. Moreover, the phosphorylation level of protein p53 was consistent with the change trend of protein NLRP3, suggesting that p53 may regulate myocardial cell apoptosis as the downstream regulatory signal of NLRP3 inflammasome.

At present, the limitation of mild hypothermia therapy in clinical application is rapid cooling and maintenance of heart temperature. One previous study has a reduced AMI area via targeted cooling in coronary arteries of isolated pig heart through PCI [36], and there are corresponding calculation models to predict the required cooling time according to the temperature and water flow speed of normal saline injected into coronary arteries [37]. Pharmacologically induced hypothermia (PIH) can avoid adverse effects of physiological feedback on patients such as shivering and vasoconstriction caused by low temperature [38]. Mild hypothermia therapy can be better applied to treat patients with AMI if its implementation problems are solved.

To sum up, this study has intervened with MI/R injury and myocardial hypoxia-reoxygenation models through mild hypothermia to explore mild hypothermia's effect on the apoptosis and inflammation level of myocardial cells and has found the protective effect of mild hypothermia therapy on myocardial cells and has also revealed that mild hypothermia may reduce the myocardial cell inflammation level and inhibit myocardial cell apoptosis by inhibiting the NLRP3 inflammasome pathway and p53 signaling pathway, which provides reliable evidence for clinical use of mild hypothermia in the treatment of patients with AMI.

## Figures and Tables

**Figure 1:** Levels of IL-6 and TNF-*α* in the serum of rat models of AMI by ELISA. (a) The serum expression of IL-6 in the four groups of rats. The IL-6 level of the IRI group was significantly increased, and the IL-6 level of the IRI + mild hypothermia group was significantly lower than that of the IRI group. (b) The serum TNF-*α* expression level of rats in the four groups. The level of TNF-*α* was significantly increased in the IRI group, and the TNF-*α* level was significantly lower in the IRI + mild hypothermia group than that in the IRI group. Mean ± SEM, *n* = 5, ^∗^*p* < 0.05 vs. sham; ^#^*p* < 0.05 vs. model.

**Figure 2:** Mild hypothermia intervention's effect on the myocardial apoptosis level and apoptotic myocardial cell count in rat models of AMI. (a) Myocardial tissue TUNEL staining pictures of rats (scale bar = 100 *μ* m). (b) Statistical chart of the myocardial tissue-stained TUNEL-positive cell count of rats. Mean ± SEM, *n* = 5; ^∗^*p* < 0.05 vs. sham; ^#^*p* < 0.05 vs. model.

**Figure 3:** Effects of mild hypothermia therapy on the phosphorylation levels of NLRP3 inflammasome and p53 in the myocardial tissue of rat models of AMI. (a) Expression of NLRP3, p-p53, and p53 in the myocardial tissue of rats according to the WB assay. (b) Histogram of gray values of NLRP3 and p-p53 in myocardial tissue of rats in each group (*n* = 5, ^∗^*p* < 0.05 vs. sham; ^#^*p* < 0.05 vs. model).

**Figure 4:** Effects of mild hypothermia on the mRNA expression of IL-6 and TNF-*α* in in vitro myocardial cell models of OGD. (a) mRNA expression of IL-6 and TNF-*α* in myocardial cells according to the PCR assay. (b) Histogram of mRNA expression of IL-6 and TNF-*α* in the myocardial tissue (*n* = 3; ^∗^*p* < 0.05 vs. control; ^#^*p* < 0.05 vs. OGD).

**Figure 5:** Mild hypothermia's effect on cell apoptosis and the inflammasome NLRP3/p53 signaling pathway of in vitro myocardial cell models of OGD. (a) Expression of NLRP3, cleaved Caspase-3, Caspase-3, p-p53, and p53 in myocardial cells in each group according to the WB assay. (b–d) The histograms of gray values of NLRP3, p-p53, and cleaved Caspase-3 in myocardial cells (*n* = 3, ^∗^*p* < 0.05 compared with control; ^#^*p* < 0.05 compared with OGD).

## Data Availability

All the raw data could be accessed by contacting the corresponding author if qualified researchers need.
